The article "Effect of Comprehensive Nursing Intervention on the Effect of CT-Guided Intravenous Thrombolysis in Acute Cerebral Infarction" was published in 2022. Journal: J Healthc Eng.

# Effect of Comprehensive Nursing Intervention on the Effect of CT-Guided Intravenous Thrombolysis in Acute Cerebral Infarction

**DOI:** 10.1155/2022/6959416

**Published:** 2022-01-17

**Authors:** Zhenzhong Sun, Hong Jiang, Cuiqing Chen, Yanxia Fan

**Affiliations:** ^1^Department of Imaging, Yantaishan Hospital, Yantai 264000, China; ^2^Department of Imaging, Yantai Yuhuangding Hospital Affiliated to Qingdao University, Yantai 26400, China; ^3^Department of Neurology (I), Affiliated Qingdao Central Hospital, Qingdao University, Qingdao 266042, China; ^4^Department of Neurology (III), The Fourth People's Hospital of Jinan, Jinan 250031, China

## Abstract

**Objective:**

To investigate the effect of comprehensive nursing intervention on the effect of CT-guided intravenous thrombolytic therapy for acute cerebral infarction.

**Methods:**

99 patients with acute cerebral infarction in the internal carotid artery system who were hospitalized in our department from December 2019 to December 2020 with an onset of 3–9 h were selected and randomly divided into two groups. All patients underwent multimode CT examinations and received rt-PA thrombolytic therapy. 52 patients with conventional care were included in the control group, and 47 patients with comprehensive nursing intervention were included in the observation group. The influence characteristics, Barthel score, serum MMP-9 level, and NIHSS score were compared between the two groups.

**Results:**

After the comprehensive nursing intervention, the total efficiency, total satisfaction, psychological status, and Barthel score of the observation group were significantly higher than those of the control group (*P* < 0.05). The serum MMP-9 level and NIHSS score were significantly lower than those of the control group (*P* < 0.05).

**Conclusion:**

The use of comprehensive nursing interventions in the CT-guided intravenous thrombolysis treatment of ACI patients reduced the degree of neurological impairment, improved the therapeutic effect, increased nursing satisfaction, and enabled better control of the condition of patients with cerebral infarction, which is worth promoting research.

## 1. Introduction

Acute cerebral infarction (ACI) is caused by stenosis of blood vessels in the neck or intracranial. There are many inducing factors, most of which are due to atherosclerosis of the aorta. Due to blocked blood supply [1–3], oxygen and other nutrients cannot adequately supply brain cells; local brain tissue will be ischemic and hypoxic necrosis, resulting in impaired neurological function [4–7]. Acute cerebral infarction is characterized by high morbidity, disability, and mortality, which seriously affects people's quality of life and poses a serious risk to human health. Statistics show that the incidence of cerebral infarction tends to be younger, and the annual incidence of cerebral infarction in young people is about 200,000. Cerebral infarction brings a heavy burden to the patient's family and society.

The article "Effect of Comprehensive Nursing Intervention on the Effect of CT-Guided Intravenous Thrombolysis in Acute Cerebral Infarction" was published in 2022. Journal: J Healthc Eng.

Currently, thrombolysis is the only treatment for acute cerebral infarction that has been proven to be the most effective by evidence-based medicine [8, 9]. Strbian et al. showed that early thrombolysis was effective in reducing the disability and mortality rates of patients with ischemic stroke, and the earlier the patients received thrombolysis, the earlier the neurological recovery and better the prognosis [10]. Currently, only 3–5% of patients with acute cerebral infarction receive intravenous thrombolysis, and many patients are lost to thrombolysis because the time of onset is unclear or the conventional time limit for thrombolysis is exceeded [11]. In thrombolytic therapy, multimode CT plays an important role, which includes CT angiography, CT perfusion imaging, and CT plain scan. The combination of the three is used to determine the penumbra tissue around cerebral infarction [12–15], which leads to safer and more effective thrombolytic therapy, and also provides an imaging basis for further expanding the time window [9, 16]. Studies have shown that the near-term efficacy and long-term prognosis of multimode CT-guided thrombolysis are significantly better than those based on the time window, and the probability of recurrent cerebral hemorrhage after thrombolysis is significantly lower [17, 18].

During intravenous thrombolytic therapy, it is also crucial to take effective care of the patient and intervene with effective nursing measures. As a scientific nursing approach, comprehensive nursing interventions are carried out according to the physical conditions of different patients and can provide more targeted nursing measures for patients with cerebral infarction. Comprehensive nursing intervention is not based on the experience of nursing staff but fully respects the main position of patients and innovates the original nursing methods to make up for the shortcomings of conventional nursing so that patients can enjoy more comprehensive scientific nursing services [19, 20]. According to clinical findings, comprehensive nursing interventions can greatly help patients' neurological functions and enable patients' physical and mental health levels to be significantly restored in a relatively short period of time.

## 2. Materials and Methods

### 2.1. Study Object

99 patients with acute cerebral infarction in the internal carotid artery system who were hospitalized in our department from December 2019 to December 2020 with an onset of 3–9 h were selected and underwent multimode CT examination (CT plain, CTA, and CTP), and 10 of them were eligible for thrombolysis and received thrombolytic therapy. All cases were treated according to the green channel care pathway developed by the thrombolytic care team. This study was approved by the ethics committee of the Fourth People's Hospital of Jinan.

The article "Effect of Comprehensive Nursing Intervention on the Effect of CT-Guided Intravenous Thrombolysis in Acute Cerebral Infarction" was published in 2022. Journal: J Healthc Eng.

### 2.2. Inclusion Criteria

Inclusion criteria were as follows: age 40–80 years; clinical symptoms conforming to the diagnostic criteria of ischemic cerebrovascular disease, onset within 3–9 h; NIHSS score between 4 and 24, symptoms lasting more than 30 min, no significant improvement of symptoms before thrombolysis; patients with MTT/CTA or CBF/CTA >20%, and the descending CBV area <1/3 of the middle cerebral artery blood supply area; patients' family members signed the informed consent.

### 2.3. Therapeutic Method

Routine blood and urine examinations, liver and kidney function, coagulation function, blood glucose, electrocardiogram, and head CT were performed in 2 groups. Two physicians in the thrombolytic group confirmed that the patient met the criteria for thrombolytic therapy. Meanwhile, the patients and their families were informed of the condition and the advantages and disadvantages of thrombolytic therapy, and informed consent was signed.

In the control group, rt-PA thrombolysis was given at a dose of 0.9 mg/kg (a maximum dose of 90 mg), and 10% of the total dose was pushed intravenously within 1 min, and then the remaining 90% was pumped intravenously at a uniform rate within 1 h. After rechecking the cranial CT 24 h after thrombolysis to exclude intracranial hemorrhage, oral aspirin 200 mg/d was administered, and routine neurological care was given. In the observation group, on the basis of the abovementioned study, oral aspirin 200 mg/d was given along with anticipatory nursing intervention. In addition to the abovementioned treatments, patients in both groups were given nerve nutrition, circulation improvement, lipid-lowering, and gastric mucosa protection treatments.

### 2.4. Prethrombolytic Care

During drug administration, the patient's pupils and consciousness were observed, blood pressure was measured for 15 min/time, the patient's blood oxygen, respiration, and skin rash were observed, and other adverse reactions and bleeding symptoms were observed, so as to take timely measures to deal with them.

### 2.5. Thrombolytic in Nursing

Firstly, after the end of thrombolysis, bed rest was required for at least 24 h. Consciousness, pupils, and vital signs were monitored once an hour, and continuous oxygenation and cardiac monitoring were performed, and the NIHSS scores of patients were evaluated at 2 h, 24 h, and 7 d after thrombolysis. A multimode CT examination was performed, and the patient was continuously observed for any bleeding symptoms. After the patient's condition was stabilized, health education was provided, and reasonable functional exercises were urged to promote the recovery of neurological function at an early stage. Secondly, good basic care was provided, including care of various tubes, skin, airway, and oral cavity, turning regularly, keeping bed sheets dry and clean, taking good limb position, timely aspiration and treatment, and keeping all kinds of tubes open. Also, a good job was done in handover work, strengthening bedside care, and advising patients to have a reasonable diet, which should be low fat, low salt, light, and easy to digest. Finally, psychological guidance was strengthened, patients were actively communicated with and helped them eliminate bad psychology through distraction, successful cases were introduced, and self-relaxation therapy was conducted.

The article "Effect of Comprehensive Nursing Intervention on the Effect of CT-Guided Intravenous Thrombolysis in Acute Cerebral Infarction" was published in 2022. Journal: J Healthc Eng.

### 2.6. Post-Thrombolytic Care

The 64-slice spiral CT of Philips was used for a conventional CT plain scan, and the area of interest of CTPI was determined according to the CT plain scan results. 40 mL of contrast agent gadodiamide injection was injected at 5mL/s through the median cubital vein indent needle with a double-barrel high-pressure syringe, followed by 20 mL normal saline at the same rate. After the contrast agent was injected for 5 s, the interested layer was scanned to obtain the time-density curve. The pseudocolor images of cerebral blood flow (CBF), blood volume (CBV), the mean transit time of the contrast agent (MTT), the peak time of the contrast agent (TTP), and other parameters were obtained by postprocessing with special perfusion CT software. The existence of ischemic penumbra was determined by the mismatch between CBF and CBV.

### 2.7. Comparison of Serum MMP-9 Levels

An MMP-9 kit was used to detect the serum MMP-9 levels in 2 groups. The serum MMP-9 levels were observed before treatment and at 1 h, 24 h, 72 h, and 7 d after treatment.

### 2.8. Self-Rating Anxiety Scale (SAS) and Self-Rating Depression Scale (SDS) Scores

A self-rating anxiety scale (SAS) and a self-rating depression scale (SDS) were used to evaluate the improvement of the psychological state of the two groups. According to the Chinese norm results of SAS, a standard score of less than 50 was considered normal; 50 to 60 was classified as mild anxiety; 61 to 70 was classified as moderate anxiety; and a score above 70 indicated severe anxiety. According to the Chinese norm, the standard cut-off value of the self-rating depression scale (SDS) was 53 points, and 53∼62 points were classified as mild depression. 63 to 72 were classified as moderate depression; a score above 72 was considered major depression.

The article "Effect of Comprehensive Nursing Intervention on the Effect of CT-Guided Intravenous Thrombolysis in Acute Cerebral Infarction" was published in 2022. Journal: J Healthc Eng.

### 2.9. NIHSS Score

Changes in the National Institutes of Health Stroke Scale neurological deficit (NIHSS) score (used to assess the degree of the neurological deficit on a scale of 0 to 42, with lower scores being better) were observed before and 1 h, 24 h, 72 h and 7 d after treatment.

### 2.10. Barthel Scores

Barthel scores of the ability scale for activities of daily living 3 months after treatment are as follows: (1) clinical cure: Barthel index 100, those who could go to work or participate in labor normally; (2) efficacy: Barthel index >90, those who could take care of themselves; (3) effective: Barthel index ≥70, the condition had improved significantly after treatment; and (4) ineffective: Barthel index <70, the condition had not improved significantly or deteriorated after treatment. Barthel scores were compared by effective rate; that is, the percentage of cured, effective, and effective cases in the total number of cases.

### 2.11. Nursing Satisfaction

A self-made questionnaire was used to record the nursing satisfaction of patients at discharge. The satisfaction was divided into very satisfied, satisfied, general, and not satisfied. The total nursing satisfaction = (very satisfied + satisfied + general) × 100%.

### 2.12. Statistical Analysis

The data were analyzed by SPSS 22.0 statistical software, and the measurement data were described in the form of mean ± standard deviation (‾*x* ± *s*). The *t*-test was used to compare the data between the two groups. The counting data were described in the form of frequency and percentage [*N* (%)], and the comparison of counting data [*N* (%)] was performed by *χ*^2^ test, *P* < 0.05 was considered statistically significant.

## 3. Results

### 3.1. Baseline Data of Study Subjects

There were 52 patients in the control group, with a male to female ratio of 3 : 1; there were 47 patients in the observation group, and the male to female ratio was 3.7 : 1. The age of the included patients ranged from 54 to 72 years. There was no significant difference in gender between the two groups (*P* > 0.05). In addition, there was no statistical significance in gender, age, hypertension, coronary heart disease, stroke history, and other general information between the two groups (*P* > 0.05). As shown in Table 1, there was no statistical difference in the general baseline data of the two groups, which were comparable.

### 3.2. Image Characteristics

Of the 99 acute stroke patients included in the current study, the baseline NCCT of 3 patients (3.03%) was assessed by the imaging interpretation team as completely normal (neither early ischemic changes nor pre-existing signs). Thirty-one patients (31.31%) showed early ischemic changes (presence of early ischemic signs, combined with or without pre-existing signs) on baseline NCCT. Seventy-two patients (72.73%) had existing signs on NCCT (but did not show early ischemic changes). Low tissue density was observed on NCCT in 8 patients (8.08%), which was the highest proportion of early ischemic changes, while middle cerebral artery high density was the rarest sign of early ischemia. Pre-existing signs were more common in this study population: 81 (81.82%) patients had mild or severe encephalopathy and 83 (83.84%) patients had leukoaraiosis (Table 2).

The article "Effect of Comprehensive Nursing Intervention on the Effect of CT-Guided Intravenous Thrombolysis in Acute Cerebral Infarction" was published in 2022. Journal: J Healthc Eng.

### 3.3. Serum MMP-9 Levels in the Control Group and the Observation Group

There was no significant difference in plasma MMP-9 levels between the two groups before thrombolytic therapy (*P* > 0.05). Serum MMP-9 level in the control group and the observation group increased significantly and presented a progressive upward trend one hour after thrombolytic therapy, and peaked at 24 hours after thrombolytic therapy, followed by a gradual decline in serum MMP-9. Serum MMP-9 levels were still higher than normal baseline levels on day 7 of thrombolytic therapy. The serum MMP-9 level in both groups was higher than the normal baseline level (88.23 ng/mL), and the differences were statistically significant (*P* < 0.05). Plasma MMP-9 in the control group was higher than that in the observation group at different time periods, the difference was statistically significant (*P* < 0.05, Figure 1).

Matrix metalloproteinases are a group of zinc-dependent proteases, and MMP-9 is one of the gelatinase groups, which plays an important role in the occurrence and development of cerebral infarction. This study found that the serum MMP-9 level in patients with cerebral infarction was significantly higher than that in the normal control group at different stages of early-onset, and the serum MMP-9 level was still significantly higher at 7 days after onset. The difference was statistically significant, suggesting that MMP-9 could be used as a biomarker for predicting cerebral infarction. The significant elevation of MMP-9 24 h after onset may be related to the activation of MMP-9 expression promoted by thrombolytic drugs.

### 3.4. Psychological Status of the Two Groups before and after Nursing

In this study, the SAS score and SDS score of patients in the two groups before nursing showed no statistical difference. After the nursing intervention, the SAS score and SDS score of patients in the observation group were significantly reduced, while the SAS score and SDS score of patients in the control group showed no significant change. After the intervention, the comparison between the two groups was statistically significant (Figure 2).

The article "Effect of Comprehensive Nursing Intervention on the Effect of CT-Guided Intravenous Thrombolysis in Acute Cerebral Infarction" was published in 2022. Journal: J Healthc Eng.

### 3.5. NIHSS Score

In this study, NIHSS scores of the observation group and the control group were significantly improved at 24 h, 72 h, and 7 d after thrombolysis compared with those before thrombolysis (*P* < 0.05), indicating that the neurologic defect function of the two groups had achieved efficacy after thrombolysis. Meanwhile, NIHSS scores of the observation group were lower than those of the control group at 24 h, 72 h, and 7 d after thrombolytic therapy, with statistically significant differences (*P* < 0.05), indicating that the thrombolytic effect of the observation group was better than that of the control group (Figure 3).

### 3.6. Barthel Score in Two Groups of Patients with Cerebral Infarction

After 3 months of treatment, the differences were statistically significant (*P* < 0.05) when comparing the treatment efficiency between the observation group and the control group. In the observation group, the effective rate was 88.46%, 1 case died, the fatality rate was 2.78%, 5 cases were ineffective, and the inefficiency was 9.62%. In the control group, the effective rate was 78.72%, 2 cases died, the fatality rate was 4.76%, 8 cases were ineffective, and the ineffective rate was 17.02% (Figure 4).

### 3.7. Nursing Satisfaction of Two Groups of Patients

Through comprehensive nursing intervention, the satisfaction of the observation group reached 96.15%, which was significantly better than that of the control group (80.85%), with a statistically significant difference (*P* < 0.05) (Figure 5).

## 4. Discussion

Acute cerebral infarction is a more serious cerebrovascular disease, and patients are only able to move off the floor after a long period of recovery training after treatment, with a poor quality of life. In recent years, rt-PA intravenous thrombolysis has become the preferred clinical treatment for ACI due to its ability to fully restore the physiological function of nerve cells and neurological function [21–23] and its remarkable clinical treatment effect [24]. In the process of thrombolytic therapy, the time window of thrombolysis can be further expanded by being guided by multimode CT, thus providing a more reliable imaging basis and thus enhancing the safety and effectiveness of thrombolytic therapy. At the same time, CT examination is less time-consuming and can significantly save the onset of thrombolysis time compared with MRI examination, so multimodality CT has good prospects for clinical application [25].

The article "Effect of Comprehensive Nursing Intervention on the Effect of CT-Guided Intravenous Thrombolysis in Acute Cerebral Infarction" was published in 2022. Journal: J Healthc Eng.

Because of the serious impairment of brain function after the onset of the disease, there are certain risks during intravenous thrombolysis treatment, and patients need to actively cooperate with the treatment during thrombolysis; otherwise, some related complications and sequelae are likely to occur [26]. Therefore, it is especially critical to make good nursing interventions during ACI treatment, which can significantly improve the efficacy and prognosis of patients. In this study, we implemented nursing interventions, including before, during, and after thrombolysis, which were performed by a thrombolytic nursing team with the collaboration of multiple people according to the clinical care pathway developed by our department. The patient's condition and signs can be monitored and thrombolysis can be observed, thus actively preventing adverse events and complications. For the patient, the coordination of all phases of care can be arranged in a rational manner, thus securing the best time window for the patient's treatment and improving the thrombolytic effect.

In this study, comprehensive nursing intervention was used for intravenous thrombolytic therapy of CT-guided acute cerebral infarction. The results showed that the observation group was given predictive nursing intervention on the basis of the control group, and the total effective rate, total satisfaction, psychological status, and Barthel score of the observation group were higher than those of the control group (*P* < 0.05). Serum MMP-9 and NIHSS scores were lower than those of the control group (*P* < 0.05), indicating that the application of comprehensive nursing intervention had significant advantages and value in the same drug conditions.

## 5. Conclusion

The comprehensive nursing intervention could greatly help the patients' neurological function and enable the patients' physical and mental health to be significantly restored in a shorter period of time. The treatment efficiency of patients in the observation group was much higher than that of patients in the control group, and the comprehensive nursing intervention could better control the condition of patients with cerebral infarction, which was conducive to the formation of a good doctor-patient relationship. In conclusion, the effect of comprehensive nursing intervention on the treatment of acute cerebral infarction with intravenous thrombolysis under the guidance of CT was worthy of promotion. However, this study should be further confirmed in a larger number of patients.

## Figures and Tables

**Figure 1:** Comparison of serum MMP-9 (ng/mL) in the control group (*n* = 52) and the observation group (*n* = 47) at different time periods. Compared with before treatment, ^*∗*^*P* < 0.05; compared with the control group after treatment, ^#^*P* < 0.05.

The article "Effect of Comprehensive Nursing Intervention on the Effect of CT-Guided Intravenous Thrombolysis in Acute Cerebral Infarction" was published in 2022. Journal: J Healthc Eng.

**Figure 2:** Comparison of SAS and SDS scores between the control group (*n* = 52) and the observation group (*n* = 47). Compared with before treatment, ^*∗*^*P* < 0.05; compared with the control group after treatment, ^#^*P* < 0.05.

**Figure 3:** Comparison of NIHSS scores between the control group (*n* = 52) and the observation group (*n* = 47) before and after treatment. Compared with before treatment, ^*∗*^*P* < 0.05; compared with the control group after treatment, ^#^*P* < 0.05.

**Figure 4:** Barthel score in the control group (*n* = 52) and the observation group (*n* = 47) of patients with cerebral infarction.

**Figure 5:** Comparison of nursing satisfaction scores between the control group (*n* = 52) and the observation group (*n* = 47).

**Table 1:** Baseline comparison between the two groups.

Variable	Control group (*n* = 52)	Observation group (*n* = 47)	*P*
Gender			0.93
Male	39 (75)	37 (78.72)	
Female	13 (25)	10 (21.28)	
Age (years) (*x* ± *s*)	63.29 ± 8.61	62.56 ± 8.25	0.31
Hypertension	43 (83)	41 (87)	0.49
Type 2 diabetes	16 (31)	15 (32)	0.72
Coronary heart disease	13 (25)	15 (32)	0.8
Dyslipidemia	41 (79)	38 (81)	0.93
A history of stroke	11 (21)	14 (30)	0.37
NIHSS score	11.5 ± 3.65	11.34 ± 3.61	0.69
Time of therapy (h)	3.5 ± 0.0	3.4 ± 0.5	0.069

**Table 2:** Image characteristics of the observation group and the control group.

Image characteristics	Control group (*n* = 52)	Observation group (*n* = 47)
Preliminary evaluation		
Completely normal	2 (3.85)	1 (2.13)
Not completely normal but there were no ischemic changes	33 (63.46)	32 (68.09)
Early ischemic changes	17 (32.69)	14 (29.79)

Early ischemia changes range		
None	37 (71.15)	35 (74.47)
≤33%	12 (23.08)	9 (19.15)
＞33%	3 (5.77)	3 (6.38)

ASPECTs scores in the middle cerebral artery region		
0–7	2 (3.85)	3 (6.38)
8–10	50 (96.15)	44 (93.62)

Degree of low density tissue		
None	44 (84.62)	37 (78.72)
Mild	7 (13.46)	8 (17.02)
Severe	1 (1.92)	2 (4.26)

Brain tissue swelling grade		
None	45 (86.54)	38 (80.85)
Mild	7 (13.46)	8 (17.02)
Severe	0 (0.00)	1 (2.13)
Hyperdense middle cerebral artery sign	3 (5.77)	5 (10.64)

Existing brain tissue changes		
Encephalopathy		
None	10 (19.23)	8 (17.02)
Mild	34 (65.38)	31 (65.96)
Severe	8 (15.38)	8 (17.02)

Leukoaraiosis		
None	8 (15.38)	8 (17.02)
Mild	31 (59.62）	26 (55.32)
Severe	13 (25.00)	13 (27.66)

## Data Availability

Data to support the findings of this study are available on reasonable request from the corresponding author.
